# Comparison of the Therapeutic Effects of Tension Band with Cannulated Screw and Tension Band with Kirschner Wire on Patella Fracture

**DOI:** 10.1155/2020/4065978

**Published:** 2020-08-25

**Authors:** Chengwu Liu, Haitao Ren, Chunyan Wan, Jianlin Ma

**Affiliations:** ^1^Department of Orthopedics, Qingdao Chengyang People's Hospital, Qingdao, China; ^2^Department of Microsurgery, Qingdao Chengyang People's Hospital, Qingdao, China; ^3^Department of Surgery, Qingdao Chengyang People's Hospital, Qingdao, China; ^4^Department of Spinal Arthrology, Qingdao Chengyang People's Hospital, Qingdao, China

## Abstract

**Background:**

Patella fracture accounts for 1% of bone injury, of which anatomical reduction is of great significance to the recovery. Tension band with cannulated screw and Kirschner wire is commonly used methods for the treatment of displaced patella fracture. However, there is still some controversy on the clinical efficacy of the two treatment methods.

**Objective:**

This study aimed at comparing the therapeutic effects of the cannulated screw and Kirschner wire tension bands on patella fracture and at providing more data basis for clinical selection of treatment methods for patella fracture.

**Methods:**

Altogether, 146 patients with displaced patella fracture admitted to our hospital from March 2016 to February 2018 were selected and divided into two groups according to the different treatment methods. Among them, 71 patients received tension band with a cannulated screw (TBWCS group) and 75 patients received tension band with Kirschner wire (TBWKW group). Two groups of patients were compared in terms of surgical treatment effect after one year of treatment, complications within six months after the operation and operation-related indexes. The pain visual analogue scale (VAS) score, knee flexion degree, Lysholm score, and Bostman score were recorded at 1, 3, 6, and 12 months after operation, and the activity of daily living scale (ADL) score was evaluated at the last follow-up.

**Results:**

During the operation of patella fracture patients, the intraoperative blood loss, hospitalization time, and knee flexion loss of patients in TBWCS group were less than those in the TBWKW group (*P* < 0.05), the starting time of postoperative functional exercise was earlier than that of patients in TBWKW group (*P* < 0.05), and the incidence rate of secondary operation was lower than that of patients in the TBWKW group (*P* < 0.05), but there was no statistical difference in the operation time, incision length, and postoperative fracture gap between the two groups. The results of curative effect analysis showed that the knee flexion, Lysholm score, and Bostman score of patients treated with tension band with cannulated screw were higher than those treated with Kirschner wire (*P* < 0.05), and VAS score was lower. Tension band with cannulated screw had a better curative effect on patella fracture (*P* < 0.05), lower complication rate (*P* < 0.05), and higher quality of life of patients (*P* < 0.05).

**Conclusion:**

Tension band with cannulated screw has a good curative effect on patella fracture, low incidence of complications, early start of postoperative functional exercise, and high quality of life.

## 1. Introduction

Patella is the largest sesamoid bone of the human body, which has the function of transmitting muscle strength during knee extension [1]. Patella fracture accounts for 1% of bone injury [2]. If not treated properly, complications such as traumatic knee arthritis and knee function limitation may occur [3, 4]. Anatomical reduction is of great significance to the recovery of the patella function.

Intraoperative fixation is a common method for the treatment of displaced patella fracture, which can better recover joint function and quadriceps femoris function, and prevent osteoarthritis [5, 6]. Traditionally, the Kirschner wire tension band method is widely used, which is superior to other surgical methods in terms of tension resistance and can recover patella function to the maximum extent [7]. However, foreign body reaction caused by Kirschner wire indwelling affects skin and tissues, such as inflammatory granulation tissue [8]. In addition, Kirschner wire loosening, bending, and the like may also be caused during knee exercise, resulting in treatment failure [9]. About 10%-20% of the patients suffered from displacement between fracture fragments, and 5% of the patients underwent two operations [10]. In view of this, medical workers made an improvement plan, namely, cannulated screw method, using a cannulated screw instead of Kirschner wire, cannulated screw can be embedded into bone tissue, causing less subcutaneous foreign body sensation, and can be used for annular binding fixation of more severely crushed fracture blocks without lacunae [11, 12]. However, a tension band with a cannulated screw will irritate the skin, and the metal tail will sometimes sting and damage the bone [13]. Therefore, there is still some controversy on the clinical efficacy of the two treatment methods.

This study compared the therapeutic effects of cannulated screw and Kirschner wire with tension band on patella fracture, providing more data basis for clinical selection of treatment methods for patella fracture.

## 2. Data and Methods

### 2.1. Research Participants

This study applied prospective analysis. Altogether, 146 patients with displaced patella fracture admitted to our hospital from March 2016 to February 2018 were selected and divided into two groups according to the different treatment methods. Among them, 71 patients received tension band with a cannulated screw (TBWCS group), and 75 patients received tension band with Kirschner wire (TBWKW group).

### 2.2. Inclusion and Exclusion Criteria

Inclusion criteria: patients were aged 30-75 years old; patients underwent anteroposterior and lateral X-ray films; patients were diagnosed as acute closed patella fracture with separation and displacement by X-ray; patients had complete medical records and follow-up data; patients signed informed consent forms and could cooperate with medical stuff to complete relevant diagnosis and treatment work. Exclusion criteria: patients with pathological, open, and comminuted fractures; patients with Rockwood classification of patella fractures in I, VI, and VII; patients with suppurative infection of joints, old fractures, severe acetabular destruction, or obvious degeneration; patients combined with fractures of other parts; patients with cardiopulmonary dysfunction and severe diabetes (fasting blood glucose greater than 10 mmol/L); patients with cognitive impairment could not cooperate with follow-up.

### 2.3. Treatment Method

Patients in the TBWCS group were treated with a tension band with a cannulated screw, while patients in the TBWKW group were treated with a tension band with Kirschner wire.

Kirschner wire tension band: the patient underwent general anesthesia and took the supine position. A midline longitudinal incision was taken on the patella, the full-thickness skin flap was raised, the fracture position was exposed, and then thorough debridement was carried out. Under the perspective of the c-arm X-ray machine, Kirschner wire was pried to replace and fix the fracture fragments, and continuous traction was carried out to maintain the correction stability. Kirschner wire with a diameter of 2 mm was used to fix it, and the joint cavity was cleaned. After the fixation, the 8-figure fixation outside the wire, the deep tissue was buckled and embedded, the joint cavity was cleaned, the drainage tube was retained, the wound was sutured, and the pressure dressing was carried out after the operation.

Tension band with cannulated screw: the patient underwent general anesthesia and took the supine position. A midline longitudinal incision was taken on the patella, the full-thickness skin flap was raised, the fracture position was exposed, then, thorough debridement was carried out. A sharp reduction clamp was carried out to temporarily fix the fracture fragments. After the finger proved that the patella joint surface was flat, two Kirschner wires with a diameter of 1.6 mm was used to longitudinally pass through the fractured patella, and the Kirschner wires were used as parallel as possible and located in the anterior 1/3 of the patella. Under the guidance of Kirschner wire, a 4.5 mm semithreaded stainless steel cannulated compression screw was screwed in. After the cannulated screw was embedded into the patella bone, the needle was pulled out. Steel wire was inserted from the screw, fixed in the shape of 8-figure, buckled, and embedded into deep tissue. The joint cavity was then cleaned, the drainage tube was retained, and the wound was sutured.

### 2.4. Follow-Up Arrangements

The patients in this study were followed up for 12 months. The patients were followed up, and the pain visual analogue scale (VAS), knee flexion, Lysholm score, and Bostman score were recorded at 1, 3, 6, and 12 months after operation, and the activity of daily living scale (ADL) score was evaluated at the last follow-up. ADL Score includes tips for assessing a resident's need for assistance with activities of daily living (ADLs). VAS score was 0-10, and the high score was closely related to the severity of the pain; Lysholm score was 0-100, and the high score was closely related to the better joint function; Bostman score was 0-30, and the high score was closely related to the better recovery of knee joint function; ADL score was 0-100, and the high score was closely related to the better quality of life of patients.

### 2.5. Observation Index

Two groups of patients were compared in terms of surgical treatment effect after one year of treatment, complication occurrence within 6 months after the operation and operation-related indexes, including operation time, incision length, fracture gap after the operation (Measurement was conducted according to CT image), intraoperative blood loss, hospitalization time (Measurement was conducted according to CT image), angle of knee flexion loss of affected limb, the start time of postoperative functional exercise, and incidence rate of secondary operation.

### 2.6. Efficacy Evaluation Criteria

(1) Markedly effective: patients had no pain in the knee joint after operation; knee joint movement was normal; imaging examination showed that bone healing was satisfactory, there was no traumatic arthritis, bursitis, and other complications. (2) Effective: the patient's knee joint movement was slightly limited after operation, and the bone healing was satisfactory by imaging examination. (3) Ineffective: none of the above curative effects have been achieved, delayed healing, or malunion of fracture occurred, and knee joint movement was limited. Total effective rate = markedly effective rate + effective rate.

### 2.7. Statistical Analysis

SPSS 19.0 (Asia Analytics Formerly SPSS China) was used to analyze the data. Measurement data were expressed by %, and the comparison of rates used *χ*^2^ test. The counting data were expressed by Mean ± standard deviation (mean ± SD). K-S was used to test whether the data conform to the normal distribution, the Wilcoxon test was used for nonnormal distribution data between the two groups. The comparison between the two groups for normal distribution data adopted *t*-test. The comparison between the two groups adopted *t*-test, the comparison at different time points adopted repeated measurement analysis of variance, and the back testing adopted the LSD test. *P* < 0.05 indicates that the difference is statistically significant.

## 3. Results

### 3.1. General Data

There were 71 patients in the TBWCS group, including 33 male and 38 female patients, with an age of (57.23 ± 8.67) years, and 75 patients in the TBWKW group, including 31 male and 44 female patients, with an age of (60.74 ± 14.82) years. There was no statistical difference in gender ratio and age between the two groups. There was no significant difference between the two groups in other data, such as body mass index and fracture causes (*P* > 0.05), see Table 1 for details.

### 3.2. Clinical Efficacy

One year after treatment, the markedly effective rate, effective rate, and ineffective rate of patients in the TBWCS group were 76.06%, 23.94%, and 0.00%, respectively, while those of patients in the TBWKW group were 65.33%, 26.67%, and 8.00%, respectively. There was no statistical difference in the markedly effective rate and effective rate between the two groups (*P* > 0.05), but the ineffective rate of patients in the TBWCS group was significantly lower than that in the TBWKW group (*P* < 0.05). (Table 2).

### 3.3. Operation Related Indicators

There was no statistical difference between the two groups in terms of operation time, incision length, and fracture gap after operation. The intraoperative blood loss, hospitalization time, and angle of knee flexion loss in patients with TBWCS were less than those in patients with TBWKW (*P* < 0.05). The starting time of the postoperative functional exercise of the TBWCS group was earlier than those of the TBWKW group, and the incidence of secondary operation was lower than those in patients with TBWKW (*P* < 0.05) (Table 3).

### 3.4. Pain Score

We evaluated the changes of VAS scores of the two groups of patients within 1 year after the operation, but we did not continue to follow up on the VAS scores because those of the two groups of patients were less than 1 point 6 months after the operation. The follow-up results showed that the VAS scores of the two groups decreased gradually with the time (*P* < 0.05). The VAS scores of the patients in the TBWCS group were lower than those in the TBWKW group at 1, 3, and 6 months after operation (*P* < 0.05) (Figure 1).

### 3.5. Knee Flexion Degree

At 1, 3, 6, and 12 months after operation, knee flexion degree of the two groups of patients gradually increased with the time (*P* < 0.05), and the knee flexion of patients in TBWCS group was higher than that of patients in TBWKW (*P* < 0.05) (Figure 2).

### 3.6. Lysholm Score

At 1, 3, 6, and 12 months after operation, the Lysholm scores of the two groups of patients gradually increased with the time (*P* < 0.05). The Lysholm scores of the patients in the TBWCS group were higher than those in the TBWKW group (*P* < 0.05) (Figure 3).

### 3.7. Bostman Score

At 1, 3, 6, and 12 months after the operation, the Bostman score of the two groups of patients gradually increased with the time (*P* < 0.05), while the Bostman score of the TBWCS group was higher than that of the TBWKW group (*P* < 0.05) (Figure 4).

### 3.8. Comparison of Complications between Two Groups of Patients

There was no significant difference in the incidence of knee joint movement limitation, traumatic arthritis, bursitis, displaced internal fixation, reduction loss, and delayed fracture healing between the two groups, but the total incidence of complications in the TBWCS group was lower than that in the TBWKW group (*P* < 0.05) (Table 4).

### 3.9. Quality of Life Assessment

There was no statistical difference in ADL scores between the two groups before the operation. Twelve months after operation, the ADL scores of patients in the TBWCS group were higher than those in the TBWKW group (*P* < 0.05) (Figure 5).

## 4. Discussion

Surgical is a common method for the treatment of displaced patella fracture, of which tension band fixation is the current treatment standard [14]. However, due to the complexity of patella fracture, there is no consistent conclusion on the best clinical treatment scheme at present. This study compared the therapeutic effects of cannulated screw tension band and Kirschner wire tension band on patella fracture and found that the cannulated screw tension band had more advantages in treatment of patella fracture, with a fast recovery of patients and low incidence of complications.

Cannulated screw tension band is an improved technique based on the Kirschner wire tension band. Theoretically, the cannulated screw tension band has the advantages of stable fixation and implant protection [15]. In a biomechanical analysis on the treatment of patella fracture with wire tension band by Lee et al. [16], a cannulated screw tension band has higher load-carrying capacity and rigidity, and can absorb higher energy. However, Wang et al. [17] showed that there was no significant difference between cannulated screw and Kirschner wire tension band in improving Iowa knee joint score of patella fracture patients. Lin et al. [18] also found that after 12 months of treatment, there was no significant difference between cannulated screws and Kirschner wire tension band in improvement of VAS score, knee joint mobility, flexion, and extension of patella fracture patients. Hoshino et al. [19] also reported that the failure rate of patella fracture fixation with a cannulated screw tension band was higher than that with the Kirschner wire tension band. The results of this study show that during the operation of patella fracture patients, the intraoperative blood loss, hospitalization time, and knee flexion loss of patients in TBWCS group were less than those in the TBWKW group, the starting time of postoperative functional exercise was earlier than that of patients in the TBWKW group, and the incidence rate of secondary operation was lower than that of patients in the TBWKW group, but there was no statistical difference in the operation time, incision length, and postoperative fracture gap between the two groups. The results of curative effect analysis showed that the knee flexion, Lysholm score, and Bostman score of patients treated with tension band with cannulated screw were higher than those treated with Kirschner wire, and VAS score was lower. Tension band with cannulated screw had a better curative effect on patella fracture, lower complication rate, and higher quality of life of patients. A meta-analysis report showed that there was no difference in the success rate of operation, operation time, fracture healing time, and the number of infections between the cannulated screw and Kirschner wire tension band in treating patella fracture, but cannulated screw tension band was superior to Kirschner wire tension band in reducing the incidence of complications [20]. In the internal fixation of patella fracture, biodegradable implants were not as effective as metal implants in the treatment of displaced patella fracture, but implant stimulation was the main reason for the second operation, and the removal rate of symptomatic implants after treatment with cannulated screw tension band was low (8%) [21]. Tan et al. [22] also reported in the study that the cannulated screw tension band had a better curative effect in the treatment of patella fracture compared with the Kirschner wire tension band, and it reduced the occurrence of pain caused by implants and implant loosening. These studies all supported our conclusion.

However, some problems need to be paid attention to when using a cannulated screw tension band to treat patella fracture. The cannulated screw placed in the operation needs to be of appropriate size and can be completely embedded into bone. The head and tail of the screw do not penetrate through the upper and lower ends of the patella, thus ensuring the action of the tension band of steel wire and reducing the friction loss between the screw and steel wire, steel wire, and patella.

To sum up, the cannulated screw tension band has a better curative effect on patella fracture, low incidence of complications, early start of postoperative functional exercise, and higher quality of life.

## Figures and Tables

**Figure 1:** Difference of VAS score between the two groups within 6 months after the operation. Repeated measurement analysis of variance showed that the VAS scores of the two groups of patients decreased gradually with time. The VAS scores of patients in the TBWCS group (*n* = 71) were lower than those in the TBWKW group (*n* = 75) at 1, 3, and 6 months after operation. ^∗^ indicates compared with the TBWCS group, *P* < 0.05.

**Figure 2:** Difference of knee flexion between the two groups within 12 months after the operation. Repeated measurement analysis of variance showed that the knee flexion of the two groups of patients gradually increased with time. The knee flexion of patients in the TBWCS group (*n* = 71) was higher than that of patients in the TBWKW group (*n* = 75). ^∗^ indicates compared with the TBWCS group, *P* < 0.05. ^#^ indicates compared with 1 month after treatment in the same group, *P* < 0.05; ^&^ indicates compared with 3 months after treatment in the same group, *P* < 0.05; ^@^ indicates compared with 4 months after treatment in the same group, *P* < 0.05.

**Figure 3:** Difference of Lysholm score between the two groups within 12 months after the operation. Repeated measurement analysis of variance showed that the Lysholm scores of the two groups of patients gradually increased with time. The Lysholm scores of patients in the TBWCS group (*n* = 71) were higher than those in the TBWKW group (*n* = 75). ^∗^ indicates compared with the TBWCS group, *P* < 0.05. ^#^ indicates compared with 1 month after treatment in the same group, *P* < 0.05; ^&^ indicates compared with 3 months after treatment in the same group, *P* < 0.05; ^@^ indicates compared with 4 months after treatment in the same group, *P* < 0.05.

**Figure 4:** Bostman score difference between the two groups within 12 months after the operation. Repeated measurement analysis of variance showed that the Bostman score of the two groups of patients gradually increased with time. The Bostman score of patients in the TBWCS group (*n* = 71) was higher than that of patients in the TBWKW group (*n* = 75). ^∗^ indicates compared with the TBWCS group, *P* < 0.05.

**Figure 5:** Quality of life assessment of two groups of patients. Repeated measurement analysis of variance showed that ADL scores of patients in the TBWCS group (*n* = 71) were higher than those in the TBWKW group (*n* = 75) 12 months after the operation. ^∗^ indicates *P* < 0.05.

**Table 1:** Comparison of general data of two groups of patients (mean ± SD; *n*, %).

	TBWCS (*n* = 71)	TBWKW (*n* = 75)	*χ* ^2^/*t*	*P*
Gender			0.392	0.531
Male	33 (46.48)	31 (41.33)		
Female	38 (53.52)	44 (58.67)		
Age (years)	57.23 ± 8.67	60.74 ± 14.82	1.734	0.085
Body mass index (kg/cm^2^)	22.49 ± 1.83	22.36 ± 1.86	0.671	0.425
Affected side			3.441	0.064
Left	44 (61.97)	35 (46.67)		
Right	27 (38.03)	40 (53.33)		
Cause of fracture			1.705	0.426
Fall injury	41 (57.75)	40 (53.33)		
Traffic accident	19 (26.76)	17 (22.67)		
Other	11 (15.49)	18 (24.00)		
AO/OTA			0.913	0.633
Transverse, middle (45-C1.1)	41 (57.75)	49 (65.33)		
Transverse, proximal (45-C1.2)	11 (15.49)	9 (12.00)		
Transverse, distal (45-C1.3)	19 (26.76)	17 (22.67)		
Underlying diseases			0.087	0.957
Hypertension	10 (14.08)	9 (12.00)		
Coronary heart disease	14 (19.72)	15 (20.00)		
Diabetes	5 (7.04)	5 (6.67)		
ASA classification			0.185	0.912
I	24 (33.80)	23 (30.67)		
II	42 (59.15)	46 (61.33)		
III	5 (7.04)	6 (8.00)		
Displaced distance of fracture fragment (mm)	4.3 ± 1.8	4.7 ± 1.7	1.381	0.169
Injury time before operation (days)	2.8 ± 1.2	3.3 ± 1.4	1.849	0.067

**Table 2:** Clinical efficacy (*N*, %).

	TBWCS (*n* = 71)	TBWKW (*n* = 75)	*χ* ^2^	*P*
Markedly effective	54 (76.06)	49 (65.33)	2.018	0.155
Effective	17 (23.94)	20 (26.67)	0.143	0.705
Ineffective	0 (0.00)	6 (8.00)	Fisher	0.028
Total efficiency	71 (100.00)	69 (92.00)	Fisher	0.028

**Table 3:** Operation related indicators (mean ± SD).

	TBWCS (*n* = 71)	TBWKW (*n* = 75)	*χ* ^2^/*t*	*P*
Operation time (min)	57.37 ± 9.83	54.87 ± 9.58	1.556	0.122
Incision length (cm)	6.24 ± 1.02	5.94 ± 1.09	1.715	0.089
Intraoperative blood loss (mL)	155.38 ± 28.37	187.47 ± 23.27	7.490	<0.001
Hospitalization time (days)	13.58 ± 3.53	14.57 ± 1.12	2.309	0.022
Start time of postoperative functional exercise (days)	32.13 ± 5.88	46.12 ± 9.02	11.035	<0.001
Fracture healing time (weeks)	10.7 ± 1.7	13.2 ± 3.1	5.995	<0.001
Angle of limb loss (angles)	10.8 ± 5.6	19.3 ± 7.2	7.932	<0.001
Fracture gap after operation			0.669	0.716
0 mm	52 (73.24)	58 (77.33)		
≤2 mm	14 (19.72)	11 (14.67)		
≥3 mm	5 (7.04)	6 (8.00)		
Secondary operation	1 (1.41)	11 (14.67)	6.832	0.009

**Table 4:** Comparison of complications of two groups of patients within 6 months after operation (*N*, %).

	TBWCS (*n* = 71)	TBWKW (*n* = 75)	*χ* ^2^	*P*
Limited knee joint movement	2 (2.82)	5 (6.67)	0.491	0.484
Traumatic arthritis	0 (0.00)	2 (2.67)	Fisher	0.497
Bursitis	0 (0.00)	1 (1.33)	Fisher	0.999
Displaced internal fixation	1 (1.41)	2 (2.67)	0.002	0.962
Reduction loss	2 (2.82)	4 (5.33)	0.122	0.728
Delayed fracture healing	1 (1.41)	3 (4.00)	0.204	0.652
Total	6 (8.45)	17 (22.67)	4.534	0.033

## Data Availability

All the data can be provided if other researchers need.
